The article "Activated Carbons From Winemaking Biowastes for Electrochemical Double-Layer Capacitors" was retracted in 2023. Reasons: no approval from the institution; concerns about the data.

# Activated Carbons From Winemaking Biowastes for Electrochemical Double-Layer Capacitors

**DOI:** 10.3389/fchem.2020.00686

**Published:** 2020-08-14

**Authors:** Lorena Alcaraz, Alberto Adán-Más, Pablo Arévalo-Cid, Maria de Fatima Montemor, Félix A. López

**Affiliations:** ^1^Centro Nacional de Investigaciones Metalúrgicas (CENIM), Consejo Superior de Investigaciones Científicas (CSIC), Madrid, Spain; ^2^Departamento Egenharia Química, Centro de Química Estrutural-CQE, Instituto Superior Técnico, Universidade de Lisboa, Lisbon, Portugal

**Keywords:** wine biowastes, biomass reuse, activated carbon, electrochemical double-layer capacitor, supercapacitors

## Abstract

Revalorizing organic biowaste is critical to achieve a full circular economy, where waste is transformed into resources. One of the main strategies is to produce activated carbons and use them as functional materials for electrochemical energy storage. In this study, winemaking wastes, bagasse (BAG), and cluster stalks (CS) were recovered and used in the preparation of activated carbons by a hydrothermal process. Then, they were chemically activated using KOH and investigated for electrochemical capacitor applications. The activation treatment resulted in microporous structures, characterized by a type I isotherm for low partial pressures (*P*/*P*_0_), and a type IV for higher pressures, as observed by Brunauer–Emmett–Teller surface analysis, with specific surfaces of 1,861 and 2,662 m^2^·g^−1^ for BAG and CS, respectively. These microporous structures were also investigated by means of scanning electron microscopy, revealing a high porous degree. Micro-Raman spectroscopy and X-ray photoelectron spectroscopy measurements displayed bands associated to disorder of the structure of the carbonaceous material. The electrochemical performance of the resulting materials was investigated for electrochemical energy storage applications, as supercapacitor electrode, in 1 M KOH aqueous electrolyte. These biowaste-derived materials displayed electrochemical double-layer capacitance, with 129 F·g^−1^ at 10 A·g^−1^ in the 0.1 to −1.0 V vs. saturated calomel electrode. For that reason, they are pin-pointed as potential negative electrodes for electrochemical double-layer supercapacitors and hybrid or asymmetric supercapacitors.

## Introduction

The increasing demographic evolution over the last century alongside the industrial development of highly populated countries, such as India or China, has led to an increased demand for raw materials. This need entails a great environmental risk associated with the overexploitation of natural resources and the release of industrial waste. Nowadays, new habits to minimize the environmental impact have emerged, including a growing interest on the use of natural and bio-based products (Sardella et al., 2015). In addition, different valorization processes of waste are being considered as a mean to generate more efficient and tailored materials.

The article "Activated Carbons From Winemaking Biowastes for Electrochemical Double-Layer Capacitors" was retracted in 2023. Reasons: no approval from the institution; concerns about the data.

In this sense, obtaining activated carbons from waste is, currently, one important goal. Practically any raw materials with high carbon content, including several wastes, may yield interesting and useful materials (Deiana et al., 2009). Various waste sources have been proposed for the preparation of activated carbon, from biodiesel (Gonçalves et al., 2019) to food processing waste (Ramón-Gonçalves et al., 2019; Senophiyah-Mary et al., 2019; Yaglikci et al., 2020) or agriculture industry residues (Ukanwa et al., 2019), all of them with great attractiveness owing to their large-scale production and low price. Winemaking-derived waste is a major issue in the wine industry, being Spain, the origin of the precursor wine used in this work, the third world producer of wine (Maicas and Mateo, 2020). Among others, a great amount of skins, seeds, and stems left are generated in the process (Mingo et al., 2016). In this sense, bagasse is the residual material obtained after the pressing of grapes to extract the must, and contains grape skin, pulp, and seeds. Cluster stalks are waste generated after the grapes are removed from their woody support.

Different methods have been used to obtain activated carbons such as carbonization/leaching (Deiana et al., 2009), pyrolysis (Rajamani et al., 2018), impregnation with several activation agents (Chen et al., 2017), demineralization (Chan et al., 2011), or extraction with organic solvent (Jiménez-Cordero et al., 2014), among others. However, these processes need high-temperature treatments, increasing the total cost of the process, and usually yield materials with low specific surface areas with limited use. To increase cost-effectiveness while improving the final properties of the resulting material, hydrothermal pre-carbonization is gaining attention for the preparation of carbon-based materials from several biowastes (Jain et al., 2016). The benefits of this process as pre-treatment of precursor biowaste are two-fold. One the one hand, it reduces the total cost of the production because hydrothermal carbonization followed by chemical activation leads to increased efficiency of the subsequent activation process. On the other hand, the two-step process improves the microstructural features of the final material and, as a result, the properties of the activated carbon can be tailored to the application.

Among all the potential uses of activated carbons, such as catalyst or catalyst support [Sadashiv Bubanale and Shivashankar, 2017], pollutant adsorption (Alguacil et al., 2018; Alcaraz et al., 2019, 2020), or hydrogen production (Tsyntsarski et al., 2015; Prabu et al., 2019), their application in energy storage as electrodes for electrochemical double-layer capacitors (EDLCs) (Chang and Zainal, 2019) has attracted an immense interest from the scientific community.

The article "Activated Carbons From Winemaking Biowastes for Electrochemical Double-Layer Capacitors" was retracted in 2023. Reasons: no approval from the institution; concerns about the data.

EDLCs store energy in the form of electrostatic charge at the electrode–electrolyte interface. Large active surface area materials are required to attain large capacitance values, and, for that reason, active carbons are generally used. In contrast to classical batteries, there is no Faradaic reaction involved, which would imply diffusion-controlled chemical reactions in the material that imply slower response. Therefore, EDLCs exhibit better power capabilities (Lei et al., 2013) and the absence of chemical reactions allows to extend their useful lifetime to over 100,000 charge–discharge cycles.

Although previous studies have reported the use of activated carbons from winemaking waste for energy storage applications (Jiménez-Cordero et al., 2014; Guardia et al., 2018, 2019), most literature focuses on their performance in two-electrode systems. Studying their performance in three-electrode systems is key to understanding their applicability in asymmetric and hybrid devices. Moreover, to the best of our knowledge, the study of electrochemical properties for this type of materials has been scarcely investigated in certain cases, without an in-depth investigation on their cycling stability or their performance at high applied currents.

In the present work, the preparation of activated carbons from both winemaking wastes, bagasse (BAG), and cluster stalks (CS), is described. Hydrothermal carbonization as pre-treatment of chemical activation is used to obtain activated carbons with improved specific surface. Textural properties, and structural and morphological characterization have been investigated by several techniques, and their applicability to electrochemical energy storage systems has been addressed. The electrochemical performance of the obtained activated carbons from winemaking wastes is investigated using 1 M KOH aqueous electrolyte.

## Materials and Methods

### Preparation of the Activated Carbons From the Biowastes

Activated carbons were generated from BAG and CS, winemaking wastes generated in the production of Albariño wine (Denomination of Origin “Rias Baixas,” Galicia, Spain). These biowastes were supplied by Mision Biológica de Galicia (CSIC). Both BAG and CS were separately ground to achieve a grain size of <2 mm. After that, aqueous suspensions of 75 g·L^−1^ were prepared. The mixtures were introduced into a high-pressure reactor at 523 K for 3 h and 30 bar. Then, the aqueous suspensions were filtered through a pressure filter, obtaining the activated carbon precursors. Finally, these were chemically activated with KOH (1:2 ratio) in a tubular oven under a N_2_ atmosphere (150 mL·min^−1^) at 1,073 K for 2 h. After cooling down to room temperature, the obtained activated carbons were washed with MilliQ water until a neutral pH was achieved. These materials are henceforward denominated BAG and CS.

The article "Activated Carbons From Winemaking Biowastes for Electrochemical Double-Layer Capacitors" was retracted in 2023. Reasons: no approval from the institution; concerns about the data.

### Physicochemical Characterization

The microporous structure of the obtained carbonaceous materials was evaluated by N_2_ adsorption. Measurements were carried out using a Micromeritics ASAP 2010 Accelerated Surface Area and Porosimetry System at 77 K. The specific surfaces were determined by analyzing the N_2_ adsorption isotherm from the Brunauer–Emmett–Teller (BET) equation (Brunauer et al., 1938) and Density Functional Theory (DFT) model (Nič et al., 2009) using a Micromeritics and Quantachrome software. The BET and DFT results were compared using Kaneko (Kaneko et al., 1992) and Dubinin (Nguyen and Do, 2001) equations. Micro-Raman measurements were carried out in a Horiba Jovin Yvon LabRAM HR800 system at room temperature. The samples were excited by a 633 nm He–Cd laser on an Olympus BX 41 confocal microscope with a × 40 objective. A charge-coupled device detector was used to collect the scattered light dispersed by a 2,400 lines mm^−1^ grating (micro-Raman) with a spectral resolution of 1.5 cm^−1^. X-ray photoelectron spectroscopy (XPS) spectra were recorded using a Fisons MT500 spectrometer equipped with a hemispherical electron analyzer (CLAM2) and a non-monochromatic Mg K_α_ X-ray source operated at 300 W. Spectra were collected at a pass energy of 20 eV (typical for high-resolution conditions). The area under each peak was calculated after subtraction of the S-shaped background and fitting the experimental curve to a combination of Lorentzian and Gaussian lines of variable proportions. Binding energies were calibrated to the C 1s peak at 285.0 eV. The atomic ratios were computed from the peak intensity ratios and reported atomic sensitivity factors. Morphological characterization was performed by scanning electron microscopy (SEM) using a JEOL JSM-7600F. For these observations, the powder samples were placed on an adhesive conductive carbon disk.

### Electrochemical Characterization

To evaluate the electrochemical properties of the activated carbons, a slurry was prepared using standard conditions reported elsewhere (Gören et al., 2015), that is, by mixing 80% of active material, 15% conductive carbon, and 5% PVDF dispersed in N-methyl-2-pyrrolidone. The slurry was impregnated on Toray Carbon Paper, which serves as conductive substrate, and then dried at 40°C for 12 h. Electrochemical performance was evaluated using 1 M KOH electrolyte in a three-electrode cell configuration. The coated carbon paper, a 2.5 × 2.5 cm^2^ platinum foil, and a saturated calomel electrode were employed as working, counter, and reference electrode, respectively. The electrochemical tests were performed in a Gamry Instruments IFC1000-07087 potentiostat. Cyclic voltammetry was performed at scan rates from 10 to 350 mV·s^−1^. Galvanostatic charge–discharge curves were obtained in the range −1.0 to 0.1 V at different specific currents (1–10 A·g^−1^). Electrochemical impedance spectroscopy (EIS) studies were performed after holding the electrode for 2,000 s open circuit potential to ensure signal stabilization, by applying a sinusoidal perturbation with 10 mV amplitude in the frequency range from 0.01 to 10^5^ Hz. Material stability was tested by continuous galvanostatic charge–discharge experiments at 10 A·g^−1^ during 5,000 cycles.

The article "Activated Carbons From Winemaking Biowastes for Electrochemical Double-Layer Capacitors" was retracted in 2023. Reasons: no approval from the institution; concerns about the data.

## Results and Discussion

### Characterization of the Activated Carbons

#### Textural Features

The textural properties of the activated carbons were assessed by N_2_ adsorption–desorption isotherms (Figure 1). For both activated carbons, the adsorbed N_2_ volume (cm^3^·g^−1^) significantly increases with the relative pressure (*P*/*P*_0_) for relative pressures below 0.1, which indicates the presence of microporosity in both samples. At higher relative pressures, hysteresis loops were found, indicating the presence of mesopores (Beltrame et al., 2018). These results reveal the presence of both micropores and mesopores. According to the IUPAC (Thommes et al., 2015), the obtained shapes correspond to type I and type IV isotherms, respectively. The volume of N_2_ adsorbed was lower for the BAG sample than for the CS sample. However, the micropore volume (Table 1) was similar for both activated carbons. The total pore volume for the BAG sample was lower than for CS (0.8 and 1.4 cm^3^·g^−1^, respectively). Also, the average pore sizes were 1.2 and 1.7 nm (lower than 2 nm in both cases), revealing that the obtained activated carbons mainly exhibit a microporous structure (Nič et al., 2009). The obtained results could indicate that the CS sample exhibits a greater number of mesopores. For this reason, the total volume of N_2_ adsorbed was the highest. Finally, the specific surface areas were calculated using the Dubinin and the BET equations. Although the BET equation shall be carefully interpreted for microporous materials, it is widely used for determining the specific surface area of porous carbons (Guardia et al., 2018). Therefore, BET surface areas are included for comparison purposes. The obtained values were 1,337 and 1,861 m^2^·g^−1^ for the BAG sample and 1,194 and 2,662 m^2^·g^−1^ for the CS sample. The calculated BET surfaces were higher than the obtained total surface areas from the Dubinin equation, which could be associated to pore sizes being higher than 1 nm. In these cases, the BET equation tends to overestimate the results, as previously reported in literature (Centeno and Stoeckli, 2010).

The article "Activated Carbons From Winemaking Biowastes for Electrochemical Double-Layer Capacitors" was retracted in 2023. Reasons: no approval from the institution; concerns about the data.

**Figure 1:** N_2_ adsorption–desorption isotherms for winemaking-derived activated carbons from bagasse (BAG) and cluster stalks (CS).

**Table 1:** Textural properties for both activated carbons obtained from the winemaking wastes.

	**BAG**	**CS**
Total pore volume (cm^2^·g^−1^)	0.8	1.4
Micropore volume (cm^2^·g^−1^)	0.7	0.9
Average micropore size (nm)	1.2	1.7
Microporous surface (m^2^·g^−1^)	1,244	1,111
Total surface area (m^2^·g^−1^)	1,337	1,194
*S*_BET_ (m^2^·g^−1^)	1,861	2,662

#### Scanning Electron Microscopy

SEM micrographs for the BAG and CS activated carbon samples (Figures 2A,B) exhibit a microporous microstructure. A large number of pores can be observed, caused by the chemical interaction between the precursor surface and the activation agent (KOH). The obtained pores were irregular and oval, like embedded deep holes typically observed after chemical activation (El-Naggar et al., 2015; Ravichandran et al., 2018). BAG images denote areas with material agglomerates, where porosity is found between these mass portions. Oppositely, images of carbon obtained from CS reveal low aggregated rates with larger porosity, which is in accordance with the results of nitrogen adsorption experiments.

**Figure 2:** SEM images for **(A)** BAG and **(B)** CS.

#### Micro-Raman Spectroscopy

Two predominant bands can be observed in the Raman spectra for CS and BAG samples (Figure 3) with peaks at around 1,350 and 1,600 cm^−1^. As previously reported for carbonaceous materials (Sfyris et al., 2017), these bands can be attributed to A_1g_ and E_2g_ modes, also known as D and G bands, respectively. The D band indicates the disorder and degree of defective structure, whereas the G band is related to the graphitization of the samples. The intensity ratio (*I*_D_/*I*_G_) can provide information about the disorder and graphitization degree of the activated carbons (Zhang et al., 2018; Yagmur et al., 2020). Furthermore, it has been reported that overlapped bands in the range 1,400–1,500 cm^−1^ can be observed for amorphous carbons (Shimodaira and Masui, 2002). For the obtained carbon-based materials, in both cases, the D band was more intense than the G band. The calculated ratio of the D and G Raman signal was 1.08 and 1.1 for BAG and CS, respectively. In addition, a broadening of the D band for CS was found. Thus, the obtained results indicate that the CS sample exhibits a higher disorder degree than BAG.

The article "Activated Carbons From Winemaking Biowastes for Electrochemical Double-Layer Capacitors" was retracted in 2023. Reasons: no approval from the institution; concerns about the data.

**Figure 3:** Raman spectra for BAG and CS activated carbons.

#### X-Ray Photoelectron Spectroscopy

XPS measurements were performed to investigate the chemical composition of the samples. Asymmetric broad photoionizations were found in both cases (Figures 4A,B). The deconvolution of the C 1s core-level spectra shows four different peaks, which can be assigned to the sp^2^ carbon bonding, C–O bonding, C=O bonding, and π−π^*^ transitions (Estrade-Szwarckopf, 2004; Jerng et al., 2011; Dwivedi et al., 2015). The binding energy values found for the main peak were 284.5 eV for BAG and 285.0 eV for CS. A slight shift toward lower binding energies was found. In addition, a difference in the width of the curve is appreciable when comparing both samples. These spectra are consistent with the presence of a main band with binding energy at 284 eV that corresponds to graphite, with a distortion of the peak, resulting from the appearance of disorder in the structure. The maximum of the CS photoionization appears at higher binding energies than the BAG sample and its width is considerably higher owing to this disorder. The obtained results reveal that the CS sample exhibits a lower graphitization degree, in good agreement with the obtained Raman results. π−π^*^ transition peaks are the result of the stacking of the graphitic portion. C–O/C=O signals exposed the presence of oxygen-containing surficial groups, which appears in carbonization processes in presence of oxygen and can only be eliminated at very high temperatures (Estrade-Szwarckopf, 2004).

**Figure 4:** Deconvolution of the C 1s core-level spectra for **(A)** BAG and **(B)** CS samples.

### Electrochemical Characterization

#### Electrochemical Double-Layer Capacitance Analysis

BAG and CS wine biowaste–derived materials have been investigated as potential electrode materials in EDLCs. Figures 5A,B displays cyclic voltammetry results of the carbon-based materials in 1 M KOH in the −1.1 to 0.15 V range for CS and in the −1.0 to 0.1 V electrochemical window for BAG at different scan rates. Both present a quasi-ideal capacitive response at low scan rates. Nonetheless, when comparing the performance of both samples at scan rates over 200 mV·s^−1^, CS displays a tilted cyclic voltammogram, associated to increased resistance whereas BAG's cyclic voltammetry maintains its shape even at the scan rate of 350 mV·s^−1^.

The article "Activated Carbons From Winemaking Biowastes for Electrochemical Double-Layer Capacitors" was retracted in 2023. Reasons: no approval from the institution; concerns about the data.

**Figure 5:** Electrochemical characterization of CS **(A,C)** and BAG **(B,D)** by cyclic voltammetry **(A,B)** and galvanostatic charge–discharge **(C,D)** at different scan rates and applied currents, respectively. **(E)** Capacitance retention of each material at different applied specific currents. **(F)** Capacitance retention after 5,000 cycles of continuous charge–discharge at 10 A·g^−1^ in 1 M KOH.

Discharge curves (Figures 5C,D) display a linear time–potential relationship in any case, as expected for a double-layer capacitance charge storage mechanism. On the one hand, BAG exhibits a capacitance of 134 F·g^−1^ at 1 A·g^−1^ and 129 F·g^−1^ at 10 A·g^−1^, which represents 96% capacitance retention when the applied current is ten-folded. On the other hand, CS has a capacitance of 95 F·g^−1^ at 1 A·g^−1^ and 86 F·g^−1^ at 10 A·g^−1^, corresponding to 90% capacitance retention at 10 A·g^−1^. Whereas, BAG has higher capacitance and better capacitance retention, CS is active in a slightly larger electrochemical window (Figure 5E). Both materials exhibit excellent capacitance retention at higher applied currents, indicating their potential for high-power applications.

#### Long-Term Stability

Capacitance retention was evaluated after 5,000 continuous charge–discharge cycles at 10 A·g^−1^ and presented in Figure 5F. CS retains ~98% of its initial capacitance, resulting in a capacitance of 84 F·g^−1^ after the electrochemical cycling stability evaluation. Alternatively, BAG has a slightly lower capacitance retention, with 120 F·g^−1^ at 10 A·g^−1^ after 5,000 cycles as compared with the initial 129 F·g^−1^, which represents 93% capacitance retention. Although CS shows slightly better performance, both materials display good capacitance retention after continuous charge–discharge, as expected for carbon-derived materials.

Table 2 presents a brief review of previously reported activated carbons obtained from winemaking wastes applied in electrochemical energy storage for comparison purposes. The results obtained in this work display comparable performance, even when high currents are applied. In addition, cycling stability is evaluated for the first time, to the best of author's knowledge, in wine biowaste-derived carbons.

**Table 2:** Comparison of obtained electrochemical results with previous work on activated carbons from winemaking waste.

**Waste**	**Treatment**	**C** **(F·g^−1^)**	**I**	**Electrolyte**	**Cycling stability** **(%)**	**References**
Grape seed	Air/O_3_/HNO_3_	90–130	200 mA·g^−1^	H_2_SO_4_ 1 M	–	Jiménez-Cordero et al., 2014
		50–70	200 mA·g^−1^	Na_2_SO_4_ 1 M	–	
		80–110	200 mA·g^−1^	KOH 1 M	–	
Grape seed	KOH	75	200 mA·cm^−2^	H_2_SO_4_	–	Guardia et al., 2019
	CO_2_	45	200 mA·cm^−2^	H_2_SO_4_	–	
Bagasse	KOH	262–268	1 mA·cm^−2^	H_2_SO_4_ 2 M	–	Guardia et al., 2018
		142	1 mA·cm^−2^	EMImBF4/AN	–	
Stalks	KOH	289–296	1 mA·cm^−2^	H_2_SO_4_ 2 M	–	
		145–179	1 mA·cm^−2^	EMImBF4/AN	–	
Grape seed	KOH	262–269	1 mA·cm^−2^	H_2_SO_4_ 2 M	–	
		157–160	1 mA·cm^−2^	EMImBF4/AN	–	
Grape seed	KOH	210–300	1 mA·cm^−2^	H_2_SO_4_ 2 M	–	Suárez and Centeno, 2020
	CO_2_	80–160	1 mA·cm^−2^	H_2_SO_4_ 2 M	–	
Bagasse	KOH	260–270	1 mA·cm^−2^	H_2_SO_4_ 2 M	–	
	CO_2_	150–160	1 mA·cm^−2^	H_2_SO_4_ 2 M	–	
Stalks	KOH	260–270	1 mA·cm^−2^	H_2_SO_4_ 2 M	–	
Bagasse (BAG)	KOH	134	1 A·g^−1^	KOH 1 M	–	This work
		129	10 A·g^−1^	KOH 1 M	93 (5,000 cycles)	This work
Stalks (CS)	KOH	95	1 A·g^−1^	KOH 1 M	–	This work
		86	10 A·g^−1^	KOH 1 M	98 (5,000 cycles)	This work

The article "Activated Carbons From Winemaking Biowastes for Electrochemical Double-Layer Capacitors" was retracted in 2023. Reasons: no approval from the institution; concerns about the data.

#### Electrochemical Impedance Spectroscopy

Figure 6 illustrates the electrochemical impedance spectroscopy results for the CS and BAG-derived materials. Both display a quasi-ideal capacitive behavior, usually observed in carbon-based materials. This is in accordance with the results obtained by cyclic voltammetry and galvanostatic discharge. At high and mid-frequencies, from 10^5^ to ~1–10 Hz, both materials display a purely resistive behavior, with a plateau in the modulus frequency (Figure 6A) and a close-to-zero phase angle (Figure 6B). The Nyquist plot (Figure 5C) shows an equivalent series resistance (ESR) of 2.65 Ohm for BAG and a charge-transfer resistance of 151 mOhm, whereas the CS-derived material displays an ESR of 3.8 Ohm and a charge-transfer resistance of 89 mOhm. Equivalent series resistance arises from the wiring and current collector resistance, the electrolyte resistance, and the contact and ionic resistances associated to the electrode–electrolyte interphase (Li et al., 2015). Both materials, prepared under the same conditions, present a depressed semi-circle, which accounts for the internal resistance of the electrode. In any case, both materials present a quasi-ideal behavior with a nearly parallel response to the imaginary axis in the mid- and low-frequency range, as observed in the Nyquist plot, and a phase angle close to −80°. Nonetheless, a deviation from the ideal behavior is explained by the contribution to the total impedance of certain diffusion-controlled phenomena that may be associated to the materials' porosity.

**Figure 6:** **(A–C)** Electrochemical impedance spectroscopy results for CS and BAG after 1 and 5,000 charge–discharge cycles. **(D)** Complex analysis of impedance results.

#### Complex Capacitance Analysis

The real and imaginary capacitances as a function of the frequency are obtained using a complex capacitance analysis (Taberna et al., 2003), as described by the following equations and presented in Figure 6D.


(1) $$\begin{array}{l} C^{\prime }\left(\omega \right)=-\frac{Z^{\prime \prime }\left(\omega \right)}{2\pi f|Z\left(\omega \right){|}^{2}} \end{array}$$

(2) $$\begin{array}{l} C^{\prime \prime }=\frac{Z^{\prime }\left(\omega \right)}{2\pi f|Z\left(\omega \right){|}^{2}} \end{array}$$

where *Z*′ and *Z*″ are the real and imaginary parts of impedance in Ohm, respectively, *f* is the frequency in Hz, and |*Z*(ω)| is the modulus of impedance in Ohm. The real part of impedance attains a value of 145 mF·cm^−2^ for BAG, whereas CS displays 88 mF·cm^−2^, in accordance with the evolution observed by means of the galvanostatic discharge curves. As observed, the imaginary part goes thought a maximum at a certain frequency (***f***_0_) that defines a time constant, known as the characteristic relaxation time constant τ_0_ = 1/***f***_0_. This is considered a supercapacitor's factor of merit and is defined as “the minimum time needed to discharge all the energy from the device with an efficiency >50%” (Pech et al., 2010). In this case, CS has a factor of merit of 3.9 s, whereas BAG displays only 1.6 s, in agreement with the ESR values and the good performance at high applied currents.

The article "Activated Carbons From Winemaking Biowastes for Electrochemical Double-Layer Capacitors" was retracted in 2023. Reasons: no approval from the institution; concerns about the data.

Finally, EIS is evaluated after the first and last discharge curve during the cycling stability test (Figure 6). Three main features can be observed after 5,000 cycles. First, there is a 10% increase in the ESR. Second, the charge-transfer resistance for CS is maintained whereas for BAG it is slightly reduced to 126 mOhm. Third, both materials present almost identical behavior at mid- and low frequencies before and after continuous cycling, with the exception of CS at frequencies below 0.5 Hz, that presents a slightly decreased phase angle to −82° and BAG at frequencies lower than 0.03 Hz, which decreases its phase angle in 2°. Considering these results altogether, the integrity of the energy storage process, correlated to the active surface and porosity of the activated carbon, is maintained through continuous charge–discharge, thus retaining most of the initial capacitance of the material, as observed in Figure 5F, but a slight increase in system resistance for BAG, probably as a result of pore clogging leading to a smaller capacitance retention than for CS. Nonetheless, both materials show excellent properties for electrochemical double layer applications.

The electrochemical performance of a material is the result of its morphological character, chemical composition, and their interaction with the electrolyte. As observed by means of N_2_ adsorption experiments, both materials present great microporous surfaces, being slightly larger for BAG. This bagasse-derived carbon also possesses higher order and graphitic nature, as revealed by Raman and XPS. Therefore, this enhanced structure and chemical composition are reflected in the final electrochemical results, leading to lowered system resistance, as observed by cyclic voltammetry and electrochemical impedance spectroscopy, affecting final capacitance and performance at higher scan rates and applied currents. All these factors result in a better electrochemical performance of BAG when compared with CS. Nonetheless, both materials present excellent performance as negative electrodes for electrochemical energy storage. Therefore, BAG and CS can potentially be reinserted in a circular economy approach after their chemical activation.

The article "Activated Carbons From Winemaking Biowastes for Electrochemical Double-Layer Capacitors" was retracted in 2023. Reasons: no approval from the institution; concerns about the data.

## Conclusions

Activated carbons were obtained from different winemaking wastes, bagasse (BAG) and cluster stalks (CS), by a hydrothermal process and subsequent chemical activation with KOH. This process leads to activated carbons with specific surfaces of 1,861 and 2,662 m^2^·g^−1^ for the BAG and CS samples, respectively. As adsorption–desorption N_2_ isotherms reveal the presence of micropores and mesopores in both samples. Raman spectra for both activated carbons exhibit two predominant bands assigned to the D and G bands, typical of carbonaceous materials. In addition, Raman measurements indicate that the CS-derived sample exhibits a higher disorder degree than BAG. The electrochemical properties of these activated carbons are studied for electrochemical double-layer capacitor applications. Capacitance values of 129 and 86 F·g^−1^ at 10 A·g^−1^ are obtained for BAG and CS, respectively, with stabilities over 90% in both cases after 5,000 cycles. These results endorse the future application of these materials as negative electrodes in electrochemical energy storage devices.

## Data Availability Statement

The raw data supporting the conclusions of this article will be made available by the authors, without undue reservation.

## Author Contributions

MM and FL conceived the study. LA, AA-M, and PA-C carried out the experiments, helped in the analyses and discussion of the results, and wrote the article. All authors contributed to the review, edit, and approval of the paper.

## Conflict of Interest

The authors declare that the research was conducted in the absence of any commercial or financial relationships that could be construed as a potential conflict of interest.
